# Construction of Multiobjective Planning Decision-Making Model of Ecological Building Spatial Layout under the Background of Rural Revitalization

**DOI:** 10.1155/2022/7021770

**Published:** 2022-08-31

**Authors:** Ying Liu, Yong-Di Long, Bo-Hai Wang, Xing She

**Affiliations:** ^1^Anhui Rural Revitalization Research Institute, Anhui, Hefei 230601, China; ^2^Wanjiang University of Technology, Maanshan 243031, China; ^3^Southeast University, Jiangxi, Yichun, China; ^4^Anhui University of Technology, Anhui, Tongcheng, China; ^5^Anhui University of Technology, Anhui, Maanshan 232001, China

## Abstract

In order to improve the spatial layout ability of ecological buildings under the background of rural revitalization, a multiobjective planning and decision-making model for the spatial layout of ecological buildings is constructed. Based on the visual impact detection of ecological building space, a three-dimensional rendering model is established. The block matrix matching and boundary contour parameter analysis methods are used to plan and design the layout boundary feature points, and the wavelet scale decomposition method is used to analyze the mixed tone of the layout image. Based on this, a multiobjective planning decision-making model for the spatial layout of ecological buildings is established, based on which the spatial layout design scheme of ecological buildings is output to realize the spatial layout planning of ecological buildings. The simulation results show that the spatial layout of ecological buildings using this method is more reasonable, and the expression ability of ecological aesthetics is stronger, which has a good application value in rural planning and design.

## 1. Introduction

Under the background of rural revitalization, the spatial layout of ecological buildings is mainly embodied in: ① Respecting nature and creating ecological beauty: traditional villages are often bred under specific natural and geographical conditions, integrating mountains, water, fields, and houses, and have a good ecological environment and beautiful pastoral scenery. The planning and design of beautiful countryside should fully respect the existing natural conditions and geographical environment, and achieve the characteristics of mountains, the style of water towns, and the taste of plains [1]. ② Perfect housing construction and create architectural beauty: the quality of the building and the reasonable layout of the building directly affect the villagers' intuitive feeling of space, and the appearance of the residential houses directly determines the external image of the village. Housing planning should be in harmony with the local situation and culture, and can reflect the regional characteristics [2]. ③ Reasonably set up the industrial layout and create a beautiful life: rural landscape is the external embodiment of rural life, and life is inseparable from production [3]. Beautiful rural landscape and reasonable industrial layout are mutually integrated and inseparable [4–6]. Once rural landscape is separated from economic production, it will become an isolated “landscape” in the eyes of villagers. The planning of beautiful countryside must be based on real life, land integration through land circulation, and achieve the purpose of intensive development of collective economy. It is of great significance to study the multiobjective planning decision model of ecological building spatial layout under the background of rural revitalization [7].

Reference [8] based on the land space planning theory of “people-oriented,” through the contradiction coordination mode of “self-existence coexistence” and “optimization balance,” and taking the maximization of the overall interests of the society as the criterion, this paper constructs the decision-making path of land space ecological restoration planning of “determining the region, clarifying interests balancing needs, preliminary judgment game multidimensional evaluation, and coordinating contradictions.” Reference [9] proposes to build the overall framework of the three-dimensional decision-making platform. With the help of the Zhengyuan three-dimensional GIS platform genius world, it realizes the integrated storage management and three-dimensional visual integrated expression of basic geography, urban geology, and underground space facility data. At the same time, according to the actual business needs, an underground space auxiliary planning platform integrating above ground and underground integrated profile analysis, large-scale building site selection analysis, underground rail transit route selection planning, and underground space suitability evaluation are studied and realized. Reference [10] constructs the main structure of high-rise buildings through workset collaboration mode and integrates different building professional models. Through BIM (building information modeling) modeling software, the three-dimensional space model of high-rise building is built, and the basic information of high-rise building is added. By dividing the internal space network nodes of high-rise buildings, the emergency evacuation objectives are determined, and the limiting factors in the process of emergency evacuation are determined. Based on reasonable assumptions, a two-level decision-making model of emergency evacuation path of high-rise buildings with the optimal emergency evacuation path and the shortest emergency evacuation time is constructed. Reference [11] takes the typical representatives of the two, “spatial equilibrium model” and “confrontation generation network” as examples, summarizes, and combs their theoretical basis, advantages and limitations, and application scenarios in urban research and practice. Urban system model is more suitable for supporting large-scale planning implementation evaluation (through counterfactual simulation) and spatial planning compilation (through scenario prediction), while artificial intelligence technology is more suitable for small-scale urban spatial form generation based on current situation cases and planning guidelines. Based on their complementary advantages, cross-scale model coupling can provide a quantifiable and interpretable scientific basis for exploring local conditions, multidimensional, and win-win urban decision-making.

In this paper, combining multiobjective planning decision-making and image visual feature fusion analysis method, the spatial layout model of ecological buildings under the background of rural revitalization is designed, and a spatial layout model of ecological buildings under the background of rural revitalization based on multiobjective planning decision-making model is proposed. The visual impact of ecological building space under the background of rural revitalization is detected by using three-dimensional multiobjective planning decision of visual space and image visual feature fusion analysis method, and the three-dimensional rendering model of ecological building space under the background of rural revitalization is established. Block matrix matching and boundary contour parameter analysis method are used to plan and design the boundary feature points of ecological building space layout under the background of rural revitalization. The wavelet scale decomposition method is used to analyze the mixed tones of ecological building spatial distribution images under the background of rural revitalization, and a multiobjective planning decision model of ecological building spatial layout is established. According to the multiobjective planning decision of ecological aesthetics and image visual feature fusion analysis method, the ecological building spatial layout design under the background of rural revitalization is carried out, and the multiobjective planning decision and image visual feature fusion analysis method are used to realize the optimization of rural three-dimensional spatial layout. Finally, the performance test is carried out by simulation experiment, which shows the superior performance of this method in promoting the optimization design of ecological building spatial layout under the background of rural revitalization.

## 2. Theoretical Method of Multiobjective Programming Decision Model

Linear programming can only solve the problem of the maximum or minimum value of a goal under a set of linear constraints. In the actual decision making, we should consider several objectives to measure the advantages and disadvantages of the scheme, in which there are primary and secondary objectives. There are maximum and minimum values. There are quantitative and qualitative ones. Some are complementary and some are opposite to each other, so it is necessary to build a multiobjective planning decision model [12, 13]. By determining a reasonable weight coefficient, it can reflect the importance of different objectives. The weighted coefficient method is used to assign a weight coefficient to each objective, and the multiobjective model is transformed into a single-objective model. In goal planning, the concept of optimal solution is not mentioned, but the concept of satisfactory solution is only mentioned, that is, the solution that can take care of each goal and satisfy the decision maker is sought, and the decision maker decides which solution to choose. Absolute constraints refer to equality constraints and inequality constraints that must be strictly met, such as all constraints of linear programming problems. Solutions that cannot meet these constraints are called infeasible solutions, so they are hard constraints and rigid constraints. The goal is unique to goal planning, and the right term of the constraint can be regarded as the goal value to be pursued [14]. When the target value is reached, positive or negative deviations are allowed. Therefore, positive and negative deviation variables are added to these constraints, which are soft constraints and flexible constraints. Positive and negative deviation variables can transform absolute constraints into flexible constraints by adding positive and negative deviation variables. The objective function of the planning method is constructed according to the positive and negative deviation variables of each objective constraint, and the corresponding priority factors and weight coefficients are given. When each target value is determined, the decision maker's requirement is to minimize the deviation from the target value. Therefore, the objective function of objective programming can only be the weighted sum of all deviation variables. According to the priority order, the objective programming problem is decomposed into a series of single-objective programming problems, and then solved in turn. All the objectives are solved one by one, and after the previous objective is solved, the result of the previous objective is taken as a rigid constraint in the solution of the later objective.

The principle of multiobjective decision making is a code of conduct that should be followed in the practice of multiobjective decision making. It mainly includes:

1. On the premise of meeting the needs of decision making, we try to reduce the number of targets. We can eliminate the subordinate targets and combine the similar targets into one target, or reduce the secondary targets that only require to meet the minimum standard but not the optimization as constraints. And through the methods of summing with the same measure, averaging or forming a comprehensive function, the purpose is achieved by using comprehensive indicators instead of single indicators.
2. decide the choice of goals according to their priorities. Therefore, it is necessary to arrange the objectives in an order according to the importance degree, and specify the importance coefficient, so as to be followed in the optimization decision making.
3. For conflicting goals, we should coordinate with the overall goal as the benchmark and strive to comprehensively consider all goals.

Therefore, this paper uses this method to carry out the following research.

## 3. Image Analysis and Preprocessing of Ecological Building Spatial Layout under the Background of Rural Revitalization

### 3.1. Image Acquisition of Three-Dimensional Spatial Layout of Ecological Building Space under the Background of Rural Revitalization

In order to realize the spatial layout and high-resolution reconstruction of ecological buildings under the background of rural revitalization, the feature analysis model of three-dimensional images of ecological buildings under the background of rural revitalization was first constructed [15], and the visual impact of ecological buildings under the background of rural revitalization was detected by using three-dimensional multiobjective planning decision of visual space and image visual feature fusion analysis method [16], and the three-dimensional rendering model of ecological buildings under the background of rural revitalization was established. Three-dimensional template matching method is used to match the three-dimensional layout and image of ecological building space and analyze the boundary contour parameters under the background of rural revitalization, and the overall structure of multiobjective planning decision model of ecological building space layout under the background of rural revitalization is obtained as shown in Figure 1.

Let the distribution matrix of pixel sequence of ecological building spatial layout image under the background of three-dimensional rural revitalization be described as follows:

(1) $$\begin{array}{c} D=\left[\begin{array}{cc} I_{x}^{2} & I_{x}I_{y}\\ I_{x}I_{y} & I_{y}^{2} \end{array}\right], \end{array}$$

wherein *I*_*x*_ is the pixel of the divided area in the *X* direction, *I*_*y*_ is the pixel of the divided area in the *Y* direction, and the Radon transformation parameter space Ε of the ecological building spatial distribution image under the background of rural revitalization is Ε={*η*=(*a*, *u*, *b*) : *a*, *b* ∈ *R*, *a* > 0, *u* ∈ *S*^*d*−1^}. Let *A*={*a*_*i*_}_*i*=1_^*N*^ scalars of spatial distribution images of ecological buildings under the background of rural revitalization with multiscale texture be the set, and the CHM expression of its order mixed tone factor is as follows:

(2) $$\begin{array}{c} \kappa^{P}\left(A\right)={\left(\sum_{i=1}^{N}a_{i}^{P}\right)}^{-1/2}\left(\sum_{i=1}^{N}a_{i}^{P+1}\right){\left(\sum_{i=1}^{N}a_{i}^{P}\right)}^{-1/2}, \end{array}$$

wherein *a*_*i*_^*P*^ is a 4×4 subarea block model parameter of ecological building spatial layout image and has the following properties:

(3) $$\begin{array}{c} s\leq t\Rightarrow \kappa^{s}\left(A\right)\leq \kappa^{t}\left(A\right),\\ \underset{P⟶+\infty }{\lim}\kappa^{P}\left(A\right)=\underset{i}{\max}a_{i},\\ \underset{P⟶-\infty }{\lim}\kappa^{P}\left(A\right)=\underset{i}{\min}a_{i}, \end{array}$$

wherein *a*_*i*_ is the random degree of pixels, *A* is the spatial distribution amplitude of ecological buildings under the background of rural revitalization, and *f* is the average gray value of images in a 3×3 pixel block area [17]. Therefore, considering the spatial distribution image *κ*^*P*^ of ecological buildings under the background of rural revitalization with multiscale texture, for any pixel, let the local neighborhood of newly added seed points along the gradient direction of its texture be *B*(*x*, *y*), and there are

(4) $$\begin{array}{c} \underset{P⟶+\infty }{\lim}\kappa_{B}^{P}\left(f\right)B\left(x,y\right)=\underset{\left(s,t\right)\in BB\left(x,y\right)}{\max}f\left(s,t\right)=\delta_{B}\left(f\right)\left(x,y\right),\\ \underset{P⟶-\infty }{\lim}\kappa_{B}^{P}\left(f\right)B\left(x,y\right)=\underset{\left(s,t\right)\in BB\left(x,y\right)}{\min}f\left(s,t\right)=\varepsilon_{B}\left(f\right)\left(x,y\right), \end{array}$$

wherein *δ* and *ε*, respectively, represent the color difference expansion and color corrosion operators of three-dimensional spatial distribution of ecological building space under the background of rural revitalization, *f*(*s*, *t*) is the coordinate system of pixel distribution area, and (*x*, *y*) is the joint probability density of three-dimensional spatial distribution of ecological building space, thereby realize that collection of the spatial distribution images of ecological building under the background of rural revitalization [18].

### 3.2. Block Matrix Matching and Boundary Contour Parameter Analysis

Block matrix matching and boundary contour parameter analysis method are used to plan and design the boundary feature points of ecological building spatial layout under the background of rural revitalization [19]. *x*(*k*),  *k*=0,1,2,…, *N* − 1 is the pixel component of ecological building spatial layout under the background of rural revitalization, and **A**={**A**_*i*_}_*i*=1_^*N*^ is *N* symmetric positive definite tensors. The definition of mother wavelet of feature scale decomposition of ecological building spatial distribution image under the background of rural revitalization is as follows:

(5) $$\begin{array}{c} \kappa^{P}\left(A\right)={\left(\sum_{i=1}^{N}A_{i}^{P}\right)}^{-1/2}\left(\sum_{i=1}^{N}A_{i}^{P+1}\right){\left(\sum_{i=1}^{N}A_{i}^{P}\right)}^{-1/2}, \end{array}$$

wherein **A**_*i*_^*P*^ is the characteristic scale of the spatial distribution image of ecological buildings under the background of rural revitalization, and the mother wavelet *κ*^*P*^(**A**) of the spatial distribution image of ecological buildings under the background of rural revitalization is positive, which can correspond to the tensor model of texture characteristic space one by one to obtain *R*, G, and B components of color image W. The specific process is shown in Figure 2.

According to the affine transformation relationship, and according to the rotation, translation, and scale invariance between pixels of ecological building spatial distribution image under the background of rural revitalization, the transformation relationship between two frames of color tone information distribution characteristic points of ecological building spatial distribution image under the background of rural revitalization with multiscale texture can be described as follows:

(6) $$\begin{array}{c} X_{t}=AX_{t-1}+t, \end{array}$$

wherein *X*=[*x*_*t*_, *y*_*t*_]^*T*^ is the cluster center representing the *X* and Y directions in the spatial distribution images of ecological buildings under the background of rural revitalization, *A* is the spectral value, and *t* is the detection reflection peak of the spatial layout images of ecological buildings. After further transformation by using invariant moments, the results of block matrix matching and boundary contour parameter analysis are as follows:

(7) $$\begin{array}{c} A\;=\;s\left[\begin{array}{cc} \cos\;\theta & -\sin\;\theta \\ \sin\;\theta & \cos\;\theta \end{array}\right],\\ t=\left[\begin{array}{c} t_{x}\\ t_{y} \end{array}\right], \end{array}$$

wherein *s* is the scaling factor of matching feature points, *θ* is the rotation angle of the image area of ecological building spatial distribution image under the background of rural revitalization with multiscale texture, and tx and ty are the horizontal displacement and vertical displacement, respectively [20]. According to the above processing, the edge contour feature detection of ecological building space under the background of rural revitalization is realized. Therefore, a three-dimensional rendering model of ecological building space under the background of rural revitalization is established, and block matrix matching and boundary contour parameter analysis are used to plan and design the boundary feature points of ecological building space layout under the background of rural revitalization.

## 4. Optimization of Three-Dimensional Spatial Layout Model of Ecological Building Space under the Background of Rural Revitalization

### 4.1. 3D Rendering Model

On the basis of detecting the visual impact of ecological building space under the background of rural revitalization by using three-dimensional multi-objective planning decision of visual space and image visual feature fusion analysis method, the image analysis and three-dimensional rendering of ecological building space under the background of rural revitalization are carried out [21]. In this paper, a spatial layout model of ecological building under the background of rural revitalization based on multi-objective planning decision model is proposed. The estimated value of the spatial distribution of ecological building under the background of rural revitalization is as follows:

(8) $$\begin{array}{c} p\left(x,y;t\right)=-\sigma \nabla u\left(x,y;t\right)=-\sigma G\left(x,y;t\right)\\ =-\sigma \left[G_{x}\left(x,y;t\right)i+G_{y}\left(x,y;t\right)j\right]. \end{array}$$

In the above formula, *i*, *j* is the unit direction vector, ∇*u*(*x*, *y*; *t*) is the image pixel gradient distribution operator, *G*(*x*, *y*; *t*) is the spatial visual feature distribution value of the extracted ecological building spatial layout image under the background of three-dimensional rural revitalization, *G*_*x*_(*x*, *y*; *t*) is the approximate three-dimensional spatial feature distribution value of the extracted ecological building spatial layout image under the background of three-dimensional rural revitalization, and *G*_*y*_(*x*, *y*; *t*) is a statistical graph binary model parameter. By sampling the ecological building spatial distribution image under the background of multiscale texture rural revitalization, the white balance deviation compensation method is adopted to obtain the tone correction constraint function of the ecological building spatial distribution image under the background of rural revitalization as follows:

(9) $$\begin{array}{c} L\left(a,b_{m}\right)=\sum_{V_{m}\in P^{\text{res}}}\sum_{V_{n}\in P^{\text{true}}}Sw_{i,j}\frac{\left|V_{m}\cap V_{n}\right|}{\left|V\right|}\log\left(\frac{\left|V\right|\left|V_{m}\cap V_{n}\right|}{\left|V_{m}\right|\left|V_{n}\right|}\right). \end{array}$$

In the formula, *S* is the *R*, *G,* and *B* components of the image segmentation of ecological building spatial layout under the background of three-dimensional rural revitalization, *w*_*i*,*j*_ is the adaptive weighting coefficient, *V*_*m*_ is the difference feature quantity between pixels, and *V*_*n*_ is the characteristic distribution variance of rural building planning. After three-level Radon scale transformation, the boundary feature points of ecological building spatial layout under the background of rural revitalization are as follows:

(10) $$\begin{array}{c} L\left(a,b_{m}\right)=\sum_{V_{m}\in P^{\text{res}}}\frac{\left|V_{m}\right|}{\left|V\right|}\log\left(\frac{\left|V_{m}\right|}{\left|V\right|}\right)+\sum_{V_{n}\in P^{\text{true}}}\frac{\left|V_{n}\right|}{\left|V\right|}\log\left(\frac{\left|V_{n}\right|}{\left|V\right|}\right). \end{array}$$

Based on Radon scale transformation, the spatial distribution image blocks of ecological buildings in each rural revitalization background are decomposed in each direction, and the amplitude of the mixed tone mapping of the image rendering is A. The multiscale Retinex algorithm is used to detect the entropy information of the spatial distribution image of ecological buildings in the three-dimensional rural revitalization background [22], and the similarity feature quantity of the spatial distribution image of ecological buildings in the three-dimensional rural revitalization background is extracted. In the real matrix, the singular value decomposition result of the spatial distribution of ecological buildings in the rural revitalization background is as follows:

(11) $$\begin{array}{c} A=USV^{\prime }\\ =U\left(\begin{array}{cc} \sum & 0\\ 0 & 0 \end{array}\right)V^{\prime },\\ U*U^{\prime }=I,\\ V*V^{\prime }=I, \end{array}$$

wherein ∑=diag(*σ*_1_, *σ*_2_,…, *σ*_*r*_),  *σ*_1_ ≥ *σ*_2_ ≥ ···≥*σ*_*r*_ > 0 is the multiscale texture information fusion feature vector of the spatial distribution image of ecological buildings in the background of rural revitalization, and *A∗A*′ is the characteristic square root of *A*′*∗A*. According to the parity quantization, the coupling coefficient of mixed tone mapping in *N* block templates is obtained

(12) $$\begin{array}{c} Aa_{i,j}=U_{i,j}*S_{i,j}*V_{i,j}^{T}, \end{array}$$

wherein *U*_*i*,*j*_ is the ambiguity coefficient of the spatial layout image of ecological buildings under the background of three-dimensional rural revitalization, *S*_*i*,*j*_ is similarity, and *V*_*i*,*j*_ is Gaussian distribution function. Wavelet scale decomposition method is used to analyze the mixed tones of the spatial distribution image of ecological buildings under the background of rural revitalization, and color difference correction and graphic rendering are carried out [23].

### 4.2. Spatial Layout Design of Ecological Buildings under the Background of Rural Revitalization

According to the multi-objective planning decision making and image visual feature fusion analysis method of ecological aesthetics, the spatial layout design of ecological buildings under the background of rural revitalization is carried out. The multi-objective planning decision making and image visual feature fusion analysis method are adopted to realize the optimization of rural three-dimensional spatial layout [24], and the wavelet scale decomposition method is adopted to analyze the mixed tones of ecological building spatial distribution images under the background of rural revitalization. The multi-objective planning decision-making model of ecological building spatial layout is established, and the image filtering model of ecological building spatial layout under the background of three-dimensional rural revitalization is constructed. The filtering function is as follows:

(13) $$\begin{array}{c} w\left(d_{ij}\right)=f\left(\left|x_{i}-x_{j}\right|\right)\\ =\frac{1}{\sqrt{2\pi }}\exp\left\{\frac{{\left(x_{i}-x_{j}\right)}^{2}}{2}\right\}, \end{array}$$

wherein *x*_*i*_ represents the filtered output of pixels on the *X* component, *x*_*j*_ represents the filtered output of ecological building spatial layout image on the *Y* component under the background of three-dimensional rural revitalization, and *f*(|*x*_*i*_ − *x*_*j*_|) represents the clustering feature quantity among pixels under the background of three-dimensional rural revitalization. The wavelet scale decomposition method is used to extract the features and map the mixed tones of the spatial distribution images of ecological buildings in the background of rural revitalization [25]. The one-dimensional wavelet transform of the spatial distribution images of ecological buildings in the background of rural revitalization with multiscale texture on the grid of the template area is as follows:

(14) $$\begin{array}{c} r_{k,l}=F_{\text{RATf}}\left(k,l\right)\\ =\frac{1}{\sqrt{N}}\sum_{\left(i,j\right)\in A_{k,l}}f\left(i,j\right), \end{array}$$

wherein *A*_*k*.*l*_ represents multiscale contour edge feature pixels, with its slope *k* and intercept *l*. The feature sets of mixed tones of ecological building spatial distribution images under the background of rural revitalization are described as *k* ∈ {0,1,2,…, *N* − 1, *N*}, *l* ∈ *A*_*N*_. The wavelet scale decomposition method is used to analyze the mixed tones of the spatial distribution images of ecological buildings under the background of rural revitalization, and the gray detection model of the spatial distribution images of ecological buildings under the background of three-dimensional rural revitalization is constructed. By using frame point matching and noise segmentation, the spectral characteristics of the detection reflection peak band of the spatial distribution images of ecological buildings under the background of three-dimensional rural revitalization are obtained as follows:

(15) $$\begin{array}{c} s\left(k\right)=\phi \cdot s\left(k-1\right)+w\left(k\right), \end{array}$$

wherein

(16) $$\begin{array}{c} \phi =\left(\begin{array}{ccccc} 1 & 0 & 0 & 0 & 0\\ 0 & 1 & 1 & 0 & 0\\ 0 & 0 & 1 & 0 & 0\\ 0 & 0 & 0 & 1 & 1\\ 0 & 0 & 0 & 0 & 1 \end{array}\right),\\ w\left(k\right)=\left(\begin{array}{c} N\left(0,\sigma_{\theta \left(k\right)}\right)\\ 0\\ N\left(0,\sigma_{x\left(k\right)}\right)\\ 0\\ N\left(0,\sigma_{y\left(k\right)}\right) \end{array}\right). \end{array}$$

In the above formula, *ϕ* is to extract the corresponding texture component, *w*(*k*) represents the deep learning weight, *s*(*k* − 1) is the distribution characteristic value of the spectral curve in the absorption valley, and *σ*_*θ*(*k*)_, *σ*_*x*(*k*)_, and *σ*_*y*(*k*)_, respectively, represent the spatial visual characteristic distribution value of the extracted ecological building spatial layout image under the background of three-dimensional rural revitalization [26]. To sum up, multi-objective planning decision and image visual characteristic fusion analysis method are adopted to optimize the rural three-dimensional spatial layout, and the implementation process of the improved algorithm is shown in Figure 3.

## 5. Simulation and Result Analysis

In order to test the application performance of this algorithm in optimizing the spatial layout of ecological buildings under the background of rural revitalization, a simulation experiment was carried out, and the simulation was established on the software platform of MATLAB R2009a. The multiobjective planning simulation structure of ecological building spatial layout is shown in Figure 4. The resolution of image acquisition of three-dimensional spatial distribution of ecological buildings under the background of rural revitalization is 15×200, the direction of image sampling is 38°, the resolution of feature reconstruction is 0.56 m, and the affine area of three-dimensional spatial layout is 500×800. See Table 1 for simulation parameter settings.

According to the above simulation environment and parameter settings, the spatial distributed design of ecological buildings under the background of rural revitalization is carried out, and the original three-dimensional spatial design is obtained as shown in Figure 5.

In this paper, the method is used to analyze the mixed tones of the spatial distribution images of ecological buildings under the background of rural revitalization, and a multiobjective planning decision model of the spatial layout of ecological buildings is established. The results of the mixed tones analysis are shown in Figure 6.

Finally, the ecological aesthetics multiobjective planning decision and image visual feature fusion analysis method are used to optimize the spatial layout of ecological buildings under the background of rural revitalization, and the optimized design effect diagram is shown in Figure 7.

From the analysis of Figure 7, it can be seen that the rationality of the spatial layout of ecological buildings is better and the expression ability of ecological aesthetics is stronger under the background of rural revitalization by using this method, which has a good application value in rural planning and design. The convergence values of multiobjective planning decision making of ecological building spatial layout under the background of rural revitalization are tested by different methods, and the comparison results are shown in Table 2.

Analysis of Table 2 shows that in 100 iterations, the convergence value of this method fluctuates between 75 and 90, the convergence value of [8] method fluctuates between 71 and 75, and the convergence value of [8] method fluctuates between 81 and 88. Therefore, the convergence value of this method is relatively higher. To sum up, this method has good convergence in the multiobjective planning decision making of ecological building spatial layout under the background of Rural Revitalization.

## 6. Conclusions

In this paper, a spatial layout model of ecological buildings under the background of rural revitalization based on multi-objective planning decision model is proposed. The visual impact of ecological building space under the background of rural revitalization is detected by using three-dimensional multiobjective planning decision of visual space and image visual feature fusion analysis method, and the three-dimensional rendering model of ecological building space under the background of rural revitalization is established. Block matrix matching and boundary contour parameter analysis method are used to plan and design the boundary feature points of ecological building space layout under the background of rural revitalization. The wavelet scale decomposition method is used to analyze the mixed tones of ecological building spatial distribution images under the background of rural revitalization, and a multiobjective planning decision model of ecological building spatial layout is established. According to the multiobjective planning decision of ecological aesthetics and image visual feature fusion analysis method, the ecological building spatial layout design under the background of rural revitalization is carried out, and the multiobjective planning decision and image visual feature fusion analysis method are used to realize the optimization of rural three-dimensional spatial layout. The research shows that the rationality of the spatial layout of ecological buildings is better and the expression ability of ecological aesthetics is stronger under the background of rural revitalization, which has a good application expression in rural planning and design.

## Figures and Tables

**Figure 1:** Multi-objective planning decision model structure of ecological building spatial layout under the background of rural revitalization.

**Figure 2:** Process of extracting (r) g and b components of color image.

**Figure 3:** Implementation process of improved algorithm.

**Figure 4:** Multiobjective planning simulation structure diagram of ecological building spatial layout under the background of rural revitalization.

**Figure 5:** Three-dimensional layout design of original ecological building.

**Figure 6:** Color tone optimization of three-dimensional spatial layout of rural ecological buildings.

**Figure 7:** Optimization design of ecological building spatial layout under the background of rural revitalization.

**Table 1:** Simulation parameter setting.

Planning sample	Statistical sample number	Edge information entropy	Equivocation	Statistical characteristics
1	3135	0.141	33.364	6.113
2	6975	0.036	5.917	1.912
3	2119	4.177	36.427	0.876
4	8901	3.812	13.091	0.394
5	2240	5.330	56.857	9.771
6	7058	7.994	8.052	4.682
7	8676	8.005	22.510	4.862
8	7134	3.905	85.661	6.863
9	8500	9.352	69.315	9.542
10	7491	4.120	10.653	6.337
11	1732	1.512	16.344	3.160
12	1316	2.380	61.151	6.203
13	1001	7.119	34.201	2.409
14	3437	4.243	60.924	4.851
15	880	8.145	50.262	0.096
16	6472	7.536	45.843	0.554
17	7825	5.766	2.291	4.574
18	4024	7.043	1.121	3.650
19	9268	3.147	0.505	0.341
20	427	0.193	0.278	5.092

**Table 2:** Convergence value of multiobjective planning decision of ecological building spatial layout under the background of rural revitalization.

Iteration steps	This method	Reference [8]	Reference [9]
10	83.52	74.49	85.02
20	78.19	72.31	82.79
30	75.71	72.30	81.76
40	79.81	73.05	83.47
50	87.43	73.98	86.65
60	85.43	72.83	85.82
70	88.48	74.54	87.09
80	80.95	73.36	83.95
90	83.14	71.56	84.86
100	81.14	72.78	84.03
110	84.48	73.55	85.42
120	89.14	73.50	87.37

## Data Availability

The raw data supporting the conclusions of this article can be obtained from the corresponding authors without undue reservation.
